This article has been retracted.

# Value of 5-Hydroxymethylcytosine in HBV-Carrying High-Risk Hepatocellular Carcinoma Population: An Evaluation Based on Differential Analysis

**DOI:** 10.1155/2022/4835417

**Published:** 2022-05-23

**Authors:** Jiao Yu, Guofeng Gao, Jing Wang, Jieqiong Zhao, Yu Zhang, Dong Jiang, Feihu Huang

**Affiliations:** ^1^Department of Infection, The Third Affiliated Hospital of Naval Military Medical University, Shanghai 200000, China; ^2^Department of Disease Prevention and Control, The Third Affiliated Hospital of Naval Military Medical University, Shanghai 200000, China; ^3^Department of Outpatient Service, The Third Affiliated Hospital of Naval Military Medical University, Shanghai 200000, China; ^4^Department of Ultrasound Clinic, The Third Affiliated Hospital of Naval Military Medical University, Shanghai 200000, China

## Abstract

**Objective:**

To clarify the application value of 5-hydroxymethylcytosine (5hmC) in evaluating the progression of chronic hepatitis B (CHB) to hepatocellular carcinoma (HCC) based on difference analysis.

**Methods:**

A total of 180 patients were enrolled. Among them, 84 patients with chronic hepatitis B virus (HBV) infection while no progression to hepatocellular carcinoma (HCC) were included in the control group (CG), and 96 patients with HCC developed from HBV infection were included in the research group (RG). Two-thirds of the samples were used in the training set and 1/3 samples in the validation set to detect the level of 5hmC in both groups based on the modified nano-hmC-Seal technique. The expression levels of 5hmC-related genes TET2 and TET3 were quantified by qPCR, and the correlation between TET3 and 5hmC was analyzed by Pearson's correlation coefficients. Receiver operating characteristic (ROC) curves were drawn to evaluate the application value of the TET3-based 5hmC prediction model in the early diagnosis of HCC.

**Results:**

(i) The expression of 5hmC in RG was lower than that in CG, no matter in the training set or the validation set. (ii) 5hmC was significantly enriched in the region between the transcription initiation site and the transcription end site but was depleted in the flanking region. (iii) 5hmC-related genes TET2 and TET3 were significantly downregulated in HCC patients, whether in the training set or the validation set. (iv) In both the training and validation sets, TET3 showed a positive association with 5hmC. (v) ROC analysis results showed that the 5hmC prediction model could be used to predict the progression of CHB to HCC (training set: AUC = 0.81, 0.729-0.893; validation set: AUC = 0.84, 0.739-0.936).

**Conclusions:**

TET3 expression based on 5hmC sequencing is a landmark molecule for evaluating the progression of HCC in CHB patients, which is worthy of further study and promotion.

## 1. Introduction

Hepatocellular carcinoma (HCC) is the most common type of primary liver cancer, with significantly increased associated mortality in recent decades [1]. Massarweh and El-Serag [2] believe that the incidence of HCC has increased nearly fourfold in the past forty years, and this trend will continue into the future. A study [3] indicates that the morbidity of HCC increased from 4.4 to 6.7 cases per 100,000 between 2000 and 2012. HCC is shown to be directly related to age and gender [4]. Chronic hepatitis B virus (HBV) infection remains the most critical risk factor for HCC, and approximately 400 million people worldwide are chronically infected with HBV, of whom a quarter will eventually develop HCC [5]. In terms of the mechanism, HBV and cyclophilin HBx interact to cause liver cell regeneration and chronic necrotizing inflammation and induce subsequent adaptive immunity and immune dysfunction, thus leading to the occurrence and development of HCC [6]. In China, the prevalence of HBV is 5%-7.99%, with 7% of the adult population over 20 years of age, indicating that China faces a potential burden related to HCC. Besides, patients with the disease still have an adverse prognosis. Therefore, improving the early diagnosis efficiency of HCC can not only reduce the risk of patients with HBV infection but also effectively improve the short-term and long-term prognosis of HCC patients.

At present, the mainstays of treatment for HCC are serum alpha-fetoprotein (AFP) and imaging examination. AFP is the most widely used serum marker for HCC in the world, whereas the deepening of research identified that many HCC patients do not show elevated AFP, which means that the clinical diagnosis of HCC (especially negative AFP) cannot rely solely on AFP [7]. As mentioned above, imaging examination also plays a crucial part in HCC screening, and the commonly used techniques include abdominal ultrasound, computed tomography (CT), and magnetic resonance imaging (MRI) [8]. However, these imaging technologies still face many open-ended problems in clinical application, as they are limited by factors such as equipment, anatomical site, operator's technical experience, and economic cost. Fortunately, the development of epigenetics in recent decades has made people realize the close relationship between DNA methylation and the pathogenesis of HCC, which indicates the potential value of DNA methylation in early diagnosis of HCC. Xu et al. [9] investigated the diagnostic and prognostic value of blood DNA methylation in HCC and found that the area under the receiver operating characteristic (ROC) curve (AUC) of DNA methylation for HCC diagnosis was 0.944 (95% CI: 0.928-0.961).

5-Hydroxymethylcytosine (5-hmC) is the first oxidation product of ten eleven translocation- (TET-) mediated 5-methylcytosine (5mC) demethylation, which is one of the important mechanisms of epigenetic regulation in mammalian biology [10]. It shows great potential value in early diagnosis and prognosis assessment of cancer. A study [11] indicates that downregulation of 5hmC is a hallmark event of poor prognosis in prostate cancer patients. As for HCC, 5hmC is also of great value in the early diagnosis of the disease as it is not only related to the clinical stage of patients but has significant tissue specificity [12]. Until this stage, the research of 5hmC in the diagnosis of HCC is still in the developmental stage. Although it has been established that 5hmC can help distinguish HCC from non-HCC patients, its application value in evaluating the likelihood of chronic hepatitis B (CHB) progressing to HCC has not been thoroughly discussed.

Accordingly, based on the modified nano-hmC-Seal technique, 5hmC modification-related genes were mined, new biomarkers were screened, and 5hmC modification was explored in this study to evaluate the risk of developing HCC in patients with CHB. The completion of this study will effectively improve the diagnostic efficiency of epigenetics in the clinical application of early HCC.

## 2. Materials and Methods

### 2.1. General Information

This study included 180 patients and divided them into a control group (CG; 84 patients with chronic HBV hepatitis) and a research group (RG; 96 HCC patients carrying HBV). In CG, there were 63 males and 21 females, with an average age of 50.69 ± 8.92 years, while in RG, the male to female ratio was 65 : 31, and the mean age was 52.10 ± 9.01 years. The two groups were not significantly different in age, sex, body mass index (BMI), aspartate aminotransferase (AST), alanine aminotransferase (ALT), carcinoembryonic antigen (CEA), and history of alcoholism and smoking (*P* > 0.05) (Table 1). All the subjects involved signed an informed consent according to the Declaration of Helsinki, and this study was approved by the Ethics Committee of the Third Affiliated Hospital of Naval Military Medical University. Two-thirds of the samples were used in the training set and one-third in the validation set.

### 2.2. Inclusion and Exclusion Criteria

Inclusion criteria for CG are as follows: male ≥ 40 and female ≥ 50; diagnosis of HBV infection by medical history and routine examinations; and no hepatitis that is caused by alcohol, drugs, HCV infection, etc. Exclusion criteria for CG are as follows: liver tumor; unstable angina, symptomatic congestive heart failure, severe arrhythmia, or myocardial infarction and prolonged QT interval (>450 ms) in the past 6 months; other malignancies within the last 5 years; and those who cannot be followed up or were engaged in other clinical trials. Inclusion criteria for RG are as follows: patients with a clear prior diagnosis of HBV who progressed to HCC. Exclusion criteria for RG are as follows: patients with hepatitis C virus or posthepatitis cirrhosis/HCC caused by other types of hepatitis.

### 2.3. 5hmC and Gene Expression Detection

After an 8-hour fasting, 1 mL of peripheral venous blood of each patient was collected. In addition, 8 mL of peripheral venous blood was collected into Roche cell-free DNA collection tubes. After thorough mixing, the blood samples were stored at 6-30°C for subsequent testing. The total free plasma DNA was extracted by ZYMO RESEARCH Quick-cfDNA Serum & Plasma kit, and the operation process strictly followed the kit instructions. 5hmC: the end of the extracted plasma free DNA was added with A, and then, the connector was added for connection and purification. Then, 5hmC labeling was carried out. Thereafter, circulating cell-free DNA (cfDNA) fragments containing 5hmC were enriched, and clean reads obtained by PCR amplification, Agilent2100 quantification, and Illumina sequencing of raw data were used as the basis for subsequent analysis. By counting the reads per gene, the sequencing errors and data volume were counted, and the sequencing quality was evaluated for library construction. The sequencing data meeting the standard were selected for Bowtie2 tool analysis. The 5hmC content per gene was determined by comparing the sequencing data with the human standard genome reference sequence. TET3 gene: TET3 gene was quantitatively analyzed by fluorescent quantitative qPCR kit and PCR instrument, and 2^-*ΔΔ*t^ was used for gene expression standardization. The relative expression of TET2 and TET3 relative to the internal reference gene GAPDH was calculated.

### 2.4. Statistical Analysis

Receiver operating characteristic (ROC) curves were drawn to evaluate the early diagnostic value of TET3 gene-based 5hmC prediction model. The experimental data were expressed as mean ± variance. Pearson's correlation analysis was used to determine the correlation between 5hmC and TET3. Independent samples *t*-test was used for statistical comparison between the two groups, and paired *t*-test was used for intragroup comparison before and after disease progression. In this study, 95% was used as the confidence interval (CI), and when *P* < 0.05, the difference was considered statistically significant. The Shapiro-Wilk test was used to determine the normal distribution of data.

## 3. Results

### 3.1. Expression of 5hmC

The expression of 5hmC in patients with chronic HBV and those with chronic HBV-carrying HCC included in this study was compared based on the modified nano-hmC-Seal technique, as shown in Figure 1. The results showed that the expression of 5hmC was significantly abundant in the region between the transcription initiation site and the transcription end site but was depleted in the flanking region. Meanwhile, in both the training set and the validation set, 5hmC was significantly lower in HCC patients than in CHB patients, with a statistical difference (training: *t* = 12.20, *P* < 0.001; validation: *t* = 5.98, *P* < 0.001).

### 3.2. Comparison of 5HMC-Related Gene Expression

In this study, the expression of 5hmC-related genes TET3 and TET2 was compared between the two groups, with results presented in Figure 2. The expression of TET3 in the training set of HCC patients was significantly lower than that in CHB patients (0.73 ± 0.21 vs. 0.98 ± 0.31), and the same was true in the validation set (0.71 ± 0.21 vs. 1.04 ± 0.27), with statistically significant differences (training: *t* = 4.39, *P* < 0.001; validation: *t* = 4.06, *P* < 0.001). As for TET2, the expression in HCC patients in the training set and the validation set was lower than that in the corresponding set of CHB patients, with statistical differences (training: *t* = 6.55, *P* < 0.001; validation: *t* = 5.36, *P* < 0.001). TET3 was selected as the gene for subsequent research. We also compared the expression of TET3 in RG before and after progression to HCC. As shown in Figure 3, in both the training set and the validation set, the serum TET3 expression decreased significantly after patients progressed to HCC (training: *t* = 13.22, *P* < 0.001; validation: *t* = 7.60, *P* < 0.001).

### 3.3. Correlation between TET3 and 5hmC

This study discussed the correlation between TET3 and 5hmC in HCC patients based on Pearson's correlation, and the results are shown in Figure 4. In both the training set and the validation set, TET3 was positively correlated with 5hmC, which indicated that the decrease of 5hmC was related to the downregulation of TET3.

### 3.4. Value of TET3-Based 5hmC Prediction Model for the Development of HCC in Patients with CHB

In this study, receiver operating characteristic (ROC) curves were plotted to evaluate the early diagnosis of HCC using the TET3-based 5hmC prediction model (Figure 5). It showed that the model can be used to assess the possibility of progression to HCC in CHB patients. The area under the ROC curve (AUC) of 5hmC in the training set was 0.81 (95% CI: 0.729-0.893), and that in the validation set was 0.84 (95% CI: 0.739-0.936), which indicates that the TET-based 5hmC prediction model can effectively diagnose HCC. In addition, the ROC curve of serum AFP in diagnosing HBV-infected HCC was analyzed. As shown in Figure 6, the AUC in the training set was 0.67 (95% CI: 0.574-0.768), and that in the validation set was 0.68 (95% CI: 0.546-0.820). The above data suggest that in evaluating the progression of HBV infection to HCC, the diagnostic efficiency of the TET3-based 5hmC prediction model is far superior to serum AFP.

## 4. Discussion

The early symptoms of HCC are relatively insidious, so once diagnosed, patients are often in the advanced stage of cancer, losing the best opportunity for treatment. Therefore, effective early diagnosis and treatment are the key to lowering the high mortality rate of HCC. However, early diagnosis of HCC is facing conundrums such as false positives, false negatives, cumbersome operation techniques, and high economic costs. With the development of epigenetics, people gradually realized the important role of 5hmC in cell biological process. Cancer diagnosis based on 5hmC level benefits from the rapid development of molecular detection methods. In this study, the modified nano-hmC-Seal technique showed high sensitivity and can accurately capture 5hmC information.

The change of DNA methylation is a hallmark event in carcinogenesis, during which epigenetic markers such as 5mC are oxidized to 5hmC under the action of TET enzyme family, thus inducing the formation and growth of malignancies in the early stage of cancer [13]. The critical role of 5hmC as a biomarker for cancer diagnosis has been increasingly documented. Guler et al. [14] studied the early diagnosis of ductal pancreatic cancer based on the enrichment degree of 5hmC in genes and found that the AUC of this model was 0.92. Xiao et al. [15] suggest that the level of 5hmC expression in cfDNA can be used to screen colorectal cancer at the early stage and participates in evaluating the potential progression of precancerous adenocarcinoma to colorectal cancer.

5hmC has potential application value for early diagnosis of HCC. One previous study [12] suggested that a predictive model constructed based on 5hmC was significantly more efficient than AFP in the early diagnosis of HCC, independent of influencing factors such as smoking or alcohol consumption. Why can the level of 5hmC be used to evaluate the progression of CHB to HCC? This may be related to the progressive loss of DNA methylation involved in 5hmC. In a chronically infected HBV transgenic mouse model [16], 5hmC is involved in DNA methylation deletion, which broke the dynamic balance between HBV methylation and demethylation, promoting a gradual increase in HBV biosynthesis. All these results suggest a close relationship between 5hmC and HBV infection. However, J. Liu et al. [17] pointed out that the decrease of 5hmC expression in HCC was associated with HBV infection. The results reported in the two preceding papers seem to be opposite. But considering that the progression of HBV infection to HCC is a complex and dynamic process, TET3 and 5hmC may not continuously increase or decrease from HBV infection to malignant tumor formation. And the present research also showed significant differences in the expression of 5hmC between patients with CHB and those with HCC. Therefore, more investigations on the mechanism are warranted.

In this study, TET2 and TET3, both 5hmC-related genes, were observed to be downregulated in HCC; and in RG, TET3 expression was significantly decreased after the patients developed HCC. In particular, this study found a significant positive correlation between TET3 and 5hmC levels in HCC. TET3 protein encoded by TET3 gene is a methylcytosine dioxygenase that mediates the molecular process of catalyzing 5mC to 5hmC [18], which just explains the correlation between TET3 and 5hmC. Thus, TET2 and TET3 are the key regulators that mediate the oxidation from 5mC to 5hmC. The reduction of 5hmC level in HCC may be attributed to the downregulation of TET2 and TET3 genes [19]. But further studies are needed to confirm the relationship between TET3 and the pathogenesis of HCC. A study [20] has confirmed that TET3 is an important link in TGF-*β* pathway regulation of liver fibrosis, which indicates that TET3 is closely related to the development of liver tissue and may participate in the carcinogenesis of normal hepatocytes. Importantly, this study identified that the TET3-based 5hmC prediction model can effectively evaluate the possibility of CHB progression to HCC, with significantly higher diagnostic efficiency than serum AFP.

## 5. Conclusion

To sum up, this study argues that TET3 expression based on 5hmC sequencing is a hallmark molecule for evaluating the progression of HCC in CHB patients. In addition, the diagnostic method based on 5hmC sequencing is noninvasive, portable, and highly sensitive, with potential value in addressing the problems of false positive, false negative, cumbersome operation technology, and high economic cost, which is worthy of further research and promotion.

## Figures and Tables

**Figure 1:** Comparison of 5hmC expression between the two groups. (a) Distribution of 5hmC in the genome. (b) Expression of 5hmC in the training set of the two groups (*t* = 12.20, *P* < 0.001). (c) Expression of 5hmC in the validation set of the two groups (*t* = 5.98, *P* < 0.001). ^∗∗∗^*P* < 0.001. HCC: hepatocellular carcinoma; CHB: chronic hepatitis B. Independent samples *t*-test was used for statistical comparison between the two groups.

**Figure 2:** Expression of 5hmC-related genes in two groups. (a) Expression of TET2 in the training set of the two groups (*t* = 4.39, *P* < 0.001). (b) Expression of TET2 in the validation set of the two groups (*t* = 4.06, *P* < 0.001). (c) Expression of TET3 in the training set of the two groups (*t* = 6.55, *P* < 0.001). (d) Expression of TET3 in the validation set of the two groups (*t* = 5.36, *P* < 0.001). ^∗∗∗^*P* < 0.001. HCC: hepatocellular carcinoma; CHB: chronic hepatitis B. Independent samples *t*-test was used for statistical comparison between the two groups.

**Figure 3:** Expression of TET3 before and after HCC diagnosis in the research group. (a) Expression of TET3 in the training group (*t* = 13.22, *P* < 0.001). (b) Expression of TET3 in the validation group (*t* = 7.60, *P* < 0.001). ^∗∗∗^*P* < 0.001. HCC: hepatocellular carcinoma. Paired sample *t*-test was used for intragroup comparison before and after disease progression.

**Figure 4:** Pearson's correlation analysis of the correlation between 5hmC and TET3. (a) Training set (*R*^2^ = 0.13, *P* < 0.001). (b) Validation set (*R*^2^ = 0.43, *P* < 0.001).

**Figure 5:** Receiver operating characteristic curve evaluation of TET3-based 5hmC prediction model. (a) Training set (AUC = 0.81, *P* < 0.001, 95% CI: 0.729-0.893). (b) Validation set (AUC = 0.84, *P* < 0.001, 95% CI: 0.739-0.936). AUC: area under curve; 95% CI: 95% confidence interval.

**Figure 6:** Diagnostic value of serum AFP in HBV-infected HCC patients assessed by receiver operating characteristic curves. (a) Training set (AUC = 0.67, *P* = 0.001, 95% CI: 0.574-0.768). (b) Validation set (AUC = 0.68, *P* = 0.015, 95% CI: 0.546-0.820). AUC: area under curve; 95% CI: 95% confidence interval.

**Table 1:** General information.

	Control group (*n* = 84)	Research group (*n* = 96)	*χ* ^2^/*t*	*P*
Age (years)	50.69 ± 8.92	52.10 ± 9.01	1.051	0.295
Gender				
Female	21	31	1.159	0.282
Male	63	65		
BMI (kg/m^2^)	20.13 ± 25	20.40 ± 1.46	1.343	0.181
History of smoking			0.182	0.669
Yes	35	37		
No	49	59		
History of alcoholism			0.930	0.335
Yes	32	30		
No	52	66		
AST (U/L)	71.41 ± 9.65	73.01 ± 11.44	1.003	0.317
ALT (U/L)	68.83 ± 7.54	67.75 ± 7.74	0.937	0.350
AFP (ng/mL)	46.05 ± 9.57	52.40 ± 9.85	4.326	<0.001
CEA (ng/mL)	20.31 ± 7.66	20.48 ± 8.11	0.139	0.890

## Data Availability

The labeled dataset used to support the findings of this study are available from the corresponding author upon request.

## Abbreviations

HCC: Hepatocellular carcinoma
HBV: Chronic hepatitis B virus
HCV: Chronic hepatitis C virus
AFP: Alpha-fetoprotein
CT: Computed tomography
MRI: Magnetic resonance imaging
ROC: Receiver operating characteristic curve
5hmC: 5-Hydroxymethylcytosine
5mC: 5-Methylcytosine
TET: Ten eleven translocation
CG: Control group
RG: Research group
BMI: Body mass index
AST: Aspartate aminotransferase
ALT: Alanine aminotransferase
CEA: Carcinoembryonic antigen
AUC: Area under curve
95% CI: 95% confidence interval.
